The article "An immunoinformatics and extensive molecular dynamics study to develop a polyvalent multi-epitope vaccine against cryptococcosis" was retracted in 2025. Reasons: unreliable results or conclusions; concerns about the peer review; concerns about the authorship.

# An immunoinformatics and extensive molecular dynamics study to develop a polyvalent multi-epitope vaccine against cryptococcosis

**DOI:** 10.1371/journal.pone.0315105

**Published:** 2024-12-31

**Authors:** Md. Razwan Sardar Sami, Nurul Amin Rani, Mohammad Mahfuz Enam Elahi, Mohammad Sajjad Hossain, Minhaz Abdullah Al Mueid, Zahidur Rahim, Rajesh B. Patil, Abu Tayab Moin, Israt Jahan Bithi, Sabekun Nahar, Israt Jahan Konika, Sneha Roy, Jannatul Aleya Preya, Jamil Ahmed

**Affiliations:** 1 Faculty of Biotechnology and Genetic Engineering, Sylhet Agricultural University, Sylhet, Bangladesh; 2 Department of Pharmacy, University of Asia Pacific, Dhaka, Bangladesh; 3 Department of Theoretical and Computational Chemistry, Faculty of Science, University of Dhaka, Dhaka, Bangladesh; 4 Department of Pharmacy, Faculty of Biological Science, Jahangirnagar University, Savar, Dhaka, Bangladesh; 5 Department of Zoology, Jahangirnagar University, Dhaka, Bangladesh; 6 Sinhgad Technical Education Societys, Sinhgad College of Pharmacy, Department of Pharmaceutical Chemistry, Pune, Maharashtra, India; 7 Department of Genetic Engineering and Biotechnology, Faculty of Biological Science, University of Chittagong, Chattogram, Bangladesh; 8 Department of Biochemistry and Chemistry, Faculty of Biotechnology and Genetic Engineering, Sylhet Agricultural University, Sylhet, Bangladesh; Cholistan University of Veterinary and Animal Sciences, PAKISTAN

## Abstract

Cryptococcosis is a lethal mycosis instigated by the pathogenic species *Cryptococcus neoformans* and Cryptococcus gattii, primarily affects the lungs, manifesting as pneumonia, and the brain, where it presents as meningitis. Mortality rate could reach 100% if infections remain untreated in cryptococcal meningitis. Treatment options for cryptococcosis are limited and and there are no licensed vaccines clinically available to treat or prevent cryptococcosis. Our study utilizes an integrated bioinformatics approaches to develop a polyvalent multiepitope subunit vaccine focusing on the key virulent proteins Heat shock transcription factor and Chaperone DnaK of both C. neoformans and C. gatti. Then in silico analysis was done to predict highly antigenic epitopes by assessing antigenicity, transmembrane topology screening, allergenecity, toxicity, and molecular docking approaches. Following this analysis, we designed two vaccine constructs integrating a compatible adjuvant and suitable linkers. These constructs exhibited notable characteristics including high antigenicity, non-toxicity, solubility, stability, and compatibility with Toll-like receptors (TLRs). The interaction between both vaccine constructs and TLR2, TLR3, and TLR9 was assessed through molecular docking analysis. Molecular dynamics simulations and MM-PBSA calculations suggest the substantial stabilizing property and binding affinity of Vaccine Construct V1 against TLR9. Both the vaccines revealed to have a higher number of interchain hydrogen bond with TLR9. These findings serve as a crucial stepping stone towards a comprehensive solution for combating cryptococcus infections induced by both *C*. *neoformans* and *C*. *gattii*. Further validation through in vivo studies is crucial to confirm the effectiveness and potential of the vaccine to curb the spread of cryptococcosis. Subsequent validation through in vivo studies is paramount to confirm the effectiveness and potential of the vaccine in reducing the spread of cryptococcosis.

## 1. Introduction

Cryptococcosis is a potentially lethal mycosis caused by diverse species within the Cryptococcus genus. The genus Cryptococcus comprises around thirty species of basidiomycetous fungus that are widely spread throughout the environment. Only two species *Cryptococcus neoformans* and *Cryptococcus gattii* are recognised as being able to infect humans [1, 2]. Diseases resulting from *C*. *neoformans* infection typically manifest in immunocompromised individuals, whereas *C*. *gattii* infection has been observed to impact immunocompetent individuals. Cryptococcal meningitis, induced by *C*. *neoformans* in immunocompromised patients, particularly those with HIV, ranks among the most prevalent life-threatening conditions. Patients infected with *C*. *gattii* often present with respiratory symptoms alongside meningoencephalitis [3, 4]. With up to a million new cases each year and a high rate of morbidity and mortality related to the infection, cryptococcal meningitis has emerged as a major worldwide health concern [1]. The onset of cryptococcal infection is initiated by the inhalation of tiny yeast cells or basidiospores produced through unisexual or heterosexual reproduction. These small infectious particles evade host defense mechanisms such as mucociliary transport, mucus trapping, and airflow turbulence upon entry into the deeper regions of the lungs [5]. During the early stages of infection, the pathogen utilizes antiphagocytic components, such capsules and melanin pigment, to fight off macrophages in the lungs. When the pathogen enters the lungs, it can cause pneumonia in people with compromised immune systems; however, in hosts with healthy immune systems, alveolar macrophages either eliminate the yeast cells or they can develop a latent infection that doesn’t cause any symptoms [6–8]. *C*. *gattii* and *C*. *neoformans* exhibit numerous characteristics that promote their ability to infect and persist within a host organism. Both species spread through the bloodstream from the lungs and passes the blood-brain barrier using various mechanisms, such as paracellular passage between endothelial cells and transcytosis through endothelial cells. Fungal infection primarily occurs through respiratory inhalation; however, fungal dissemination to the central nervous system (CNS) can cause severe meningoencephalitis, which can be fatal or leave long-term neurological consequences like motor deficits, memory loss, speech and hearing difficulties, and visual impairments [9–11]. *C*. *neoformans*, characterized by its encapsulated structure, is found ubiquitously worldwide. It exhibits a critical health risk, leading to considerable sickness and death, with approximately 1 million infections and 180,000 deaths documented annually [12]. An estimated 250,000 people worldwide are affected by cryptococcal meningitis each year, which leads to 181,000 deaths. These infections have 100% fatality rates if proper treatment is not given [13]. The genome of *C*. *neoformans* is 20 Mb in size with 14 chromosomes. It is anticipated to contain 6,574 genes, with distinct characteristics such as antisense messages accounting for 0.8% and a significant proportion of alternatively spliced genes, which make up 4.3% of the total [14]. *C*. *gattii* is predominantly distributed in tropical and subtropical regions worldwide, commonly observed residing on specific trees and within soil ecosystems. Most of the strains within these species complexes are haploid, with genomes ranging in size from around 16 to 19 Mb with approximately 14 chromosomes, along with a bipolar mating system. Cryptococcal meningitis is the medical terminology for brain infections brought on by *C*. *gattii*, which can have disastrous consequences [15, 16].

The options for treating cryptococcal meningoencephalitis (CM) are limited and often unsatisfactory because of increasing drug resistance, the high toxicity of antifungal drugs, and the poor permeability of the blood-brain barrier. High death rates of up to 15% and recurrence rates of 30–50% are frequently associated with unsuccessful medical treatments [17–19]. As of right now, there are no licensed vaccinations that can be used in clinical practice to treat or prevent cryptococcosis. The need for further research aimed at developing a potent vaccine is important due to the substantial morbidity and death associated with cryptococcosis [5, 20, 21]. Considering the aforementioned, the current work uses bioinformatics-based techniques to specifically design a multiepitope subunit vaccine targeting the key proteins, Heat shock transcription factor and chaperone DnaK. Heat shock protein modulates the expression of genes connected to the electron transport chain and TCA cycle. Both the Heat shock transcription factor and Chaperone DnaK act as a virulence factor for Cryptococcus [22, 23]. There is no proposed epitope-based polyvalent vaccine for cryptococcosis that will provide broad range protection against both C. neoformans and C. gattii at the same time. A promising approach to more efficient vaccine design is immunoinformatics, which can address challenges with different antigenic variants, individualized vaccination requirements, and newly emerging and recurring health issues. We aim to pave the way for an integrated answer to the problems of cryptococcus and other fungal infections by developing a polyvalent multiepitope subunit vaccine targeting critical proteins.

## 2. Results

### 2.1. Strain and protein selection with biophysical property analyses

The target protein sequences in FASTA format were obtained from the UniProt database. The UniProt accession numbers of the chosen protein sequences are listed in Table 1. As stated in S1 Table in S1 File, every protein that was chosen was highly antigenic, stable, and had favourable physicochemical characteristics.

**Table 1:** List of the proteins used in this study with their UniProt accession numbers.

Species	Name of the protein	UniProt accession no.
*Cryptococcus neoformans*	Chaperone DnaK	J9VPF5
	Heat shock transcription factor	J9VHZ9
*Cryptococcus gattii*	Chaperone DnaK	A0A0D0TT31
	Heat shock transcription factor	A0A0D0UXX3

### 2.2. Epitope mapping for vaccine construction

The process of developing vaccines involved predicting T-cell and B-cell epitopes and evaluating their physicochemical properties. Following that, the epitopes were evaluated for high antigenicity, non-allergenicity, non-toxicity, and high conservancy. In this instance, only those who fulfilled these requirements were chosen. Furthermore, HTL epitopes were assessed for their capacity to elicit cytokines; those that were able to perform so for at least one cytokine were incorporated into the vaccine. A list of potential CTL, HTL, and LBL epitopes is presented in S2–S4 Tables in S1 File. Eight CTL, eight HTL, and eight LBL epitopes were ultimately selected for vaccine development in accordance with the strict standards listed in S5 Table in S1 File. S6 Table in S1 File lists the tools and servers utilized for epitope screening, as well as the screening parameters. The epitopes were conjugated using particular adjuvants and linkers, and the vaccine construct underwent extensive testing to verify their high antigenicity, non-allergenicity, and non-toxicity. Illustrations of vaccine constructs 1 and 2 are shown schematically and constructively in Fig 1A and 1B.

**Fig 1:** Schematic (A) and Constructive (B) representation of vaccine construct 1 and vaccine construct 2.

### 2.3. Analyses of the biophysical and structural properties of the vaccine

Biophysical investigations revealed that vaccine constructs 1 and 2 exhibited favorable properties such as solubility, stability, and appropriateness for further investigation (refer to the Table 2). The random coil became apparent to be a predominant structure in the vaccine constructs by secondary structure analysis. Following that, the vaccine constructions’ 3D structures were created and later improved and verified. In contrast to their Z scores of -5.50 and -5.85, respectively, vaccine constructs-1 and 2 had ERRAT values of 96.744 and 96.190. The majority of residues for both vaccine designs (92.0% for vaccine construct-1 and 93.1% for vaccine construct-2) were found to be in the preferred region, according to the Ramachandran plot. Both the Vaccine construct showed excellent theoretical Isoelectric point (9.63 and 9.92), Aliphatic index (56.26 and 64.09), GRAVY (-0.419 and -0.376), and other attributes, according to the physicochemical property assessment. It was evident from the vaccines’ general biophysical and structural properties that both vaccine constructions have advantageous attributes. S1 and S2 Figs in S1 File represent the 3D model and verification of both vaccine designs while S7 Table in S1 File and S3 Fig in S1 File include more details on the secondary structure of the vaccine constructs.

**Table 2:** Antigenicity, allergenecity, solubility, and biophysical properties of vaccine construct 1 (V1) and vaccine construct 2 (V2).

Features	V1	V2
**Antigenicity**	2.0334	1.8471
**Allergenicity**	Non-Allergen	Non-Allergen
**Solubility**	0.820 (Soluble)	0.809 (Soluble)
**Number of amino acids**	243	247
**Theoretical Isoelectric point (pI)**	9.63	9.92
**Formula**	C_1008_H_1636_N_308_O_328_S_8_	C_1055_H_1728_N_320_O_326_S_8_
**Total number of atoms**	3288	3437
**(Asp + Glu)**	18	16
**(Arg + Lys)**	32	36
**Half-life**	30 hours (mammalian reticulocytes, in vitro). >20 hours (yeast, in vivo). >10 hours (Escherichia coli, in vivo).	30 hours (mammalian reticulocytes, in vitro). >20 hours (yeast, in vivo). >10 hours (Escherichia coli, in vivo).
**Aliphatic index**	56.26	64.09
**Instability index**	27.67	30.82
**GRAVY**	-0.419	-0.376

### 2.4. Disulfide engineering of vaccine constructs

The capacity to generate disulfide bonds has been found in a total of 32 pairs of amino acid residues for vaccine construct-1 and 29 pairs of amino acid residues for vaccine construct-2, employing the DbD2 server. Five pairs of amino acid residues for vaccine construct 1 (CYS 11 –CYS 40, ALA 56 –ALA 169, TYR 102 –GLY 189, SER 108- GLY 114 and ARG 161 –GLY 186) and seven pairs of residue for vaccine construct 2 (GLY 1 –ASN 4, CYS 11 –CYS 40 and ARG 43 –GLU 46, ALA 64 –ARG 70, ASP 96 –THR 99, GLY 104 –VAL 119 and LEU 216 –SER 237) were carefully selected because they were compatible with standard disulfide bond formation conditions, with energy levels less than 2.2 Kcal/mol. (S4 and S5 Figs in S1 File).

### 2.5. Molecular docking analyses

To evaluate the binding intensities of both vaccine designs with TLR2, TLR3, and TLR9, molecular docking analysis was performed. The findings revealed that vaccine design 1 had a considerably greater free binding energy and a better docking score with both TLR2 and TLR9. Vaccine construct 2 showed great binding affinity towards TLR3. Table 3 represents the docking scores acquired from the ClusPro and HDOCK servers and Fig 2 depicts the vaccine-TLR complex with respective docking energy. S6 Fig in S1 File represents the interactive residue of vaccine-TLR complex generated via Pymol software. On the basis of the assigned docking score, solubility, and other required parameters, both vaccine designs were chosen for further Molecular Dynamics simulations with the Gromacs 2020.4 package in order to assess their interaction with TLR2, TLR3, and TLR9.

**Fig 2:** The best docked complex with their respective docking energy. (A) V1-TLR9 complex (B) V2-TLR9 complex (C) V1-TLR3 complex (D) V2-TLR3 complex.

**Table 3:** Binding affinity between vaccine molecules and TLRs by ClusPro and HDOCK server.

TLR	Vaccine	ClusPro Docking Score (Kcal/mol)	HDOCK Docking Score (Kcal/mol)
TLR2 (TLR ID: 2z80)	V1	-921.9	-286.88
	V2	-918.9	-263.38
TLR3 (TLR ID: 2a0z)	V1	-1019.2	-306.03
	V2	-1040.1	-288.66
TLR9 (TLR ID: 3wpf)	V1	-1245.5	-301.04
	V2	-992.1	-297.61

### 2.6. Molecular dynamics studies

#### 2.6.1. Root mean square deviation evaluation

The RMSD in the TLR and vaccine construct chains was analyzed independently. In the case of the TLR3-vaccine construct V1 complex, the RMSD in TLR3 showed considerable deviations with an average of 0.3186 nm (Fig 3A, Table 4). The bound vaccine construct V1 showed a significantly higher RMSD with an average of 0.6079 nm. The TLR3 in the TLR3-vaccine construct V2 complex showed significantly higher RMSD with an average of 0.4152 nm, while the vaccine construct V2 had slightly lower RMSD with an average of 0.5722 nm. In both the TLR3 vaccine complexes, the RMSD in TLR3 deviated significantly throughout the simulation period. Whereas significantly lower deviations were observed in the case of TLR9 complexes, where the average RMSDs in TLR9 with V1 and V2 were 0.3955 and 0.4288 nm, respectively. The deviations in RMSD in TLR9 almost remained stable. However, slightly higher RMSDs were observed in the vaccine constructs V1 and V2 with averages of 0.6752 and 0.6278 nm, respectively.

**Fig 3:** The analysis of RMSD, RMSF, and Rg. A) RMSD in TLR3 and TLR9 (left side panel) and RMSD in vaccine constructs V1 and V2 (right side panel), B) RMSF in side chain atoms of TLR3 (left side panel), TLR9 (right side panel), C) RMSF in side chain atoms of vaccine construct V1 and vaccine construct V2, D) Radius of gyration in TLR3 and TLR9 (left side panel) and RMSD in vaccine constructs V1 and V2 (right side panel).

**Table 4:** Estimates of averages for different MDS analysis parameters.

Complex	Average (nm)			
	RMSD in backbone atoms	RMSF	Gyrate	Hydrogen bonds
**TLR3-Vaccine construct V1 complex**				
TLR3	0.3186 (0.0640)	0.1710 (0.0715)	3.3810 (0.0445)	9.24 (2.20)
V1	0.6079 (0.0772)	0.2927 (0.1481)	2.1270 (0.0353)	
**TLR3-Vaccine construct V2 complex**				
TLR3	0.4152 (0.0909)	0.1613 (0.0655)	3.2930 (0.0457)	8.65 (2.42)
V2	0.5722 (0.0788)	0.3067 (0.1674)	1.9325 (0.0350)	
**TLR9-Vaccine construct V1 complex**				
TLR9	0.3955 (0.0378)	0.1627 (0.0852)	3.2892 (0.0145)	19.28 (2.62)
V1	0.6752 (0.0676)	0.2867 (0.1636)	2.2665 (0.0415)	
**TLR9-Vaccine construct V2 complex**				
TLR9	0.4288 (0.0493)	0.2024 (0.1154)	3.3619 (0.0187)	12.70 (2.54)
V2	0.6278 (0.0660)	0.3192 (0.2351)	2.1114 (0.0527)	

Standard deviations in average values are given in parentheses.

#### 2.6.2. Root mean square fluctuation evaluation

Root mean square fluctuations (RMSF) analysis for TLR3 vaccine construct complexes showed that the TLR3 bound to vaccine construct V1 and V2 have average RMSF of 0.1710 and 0.1613 nm, respectively (Fig 3B). Meanwhile, the RMSF in V1 and V2 bound vaccines was 0.2927 and 0.3067 nm, respectively (Fig 3C). The side chain atoms of residues in the range 50 to 100 and 160 to 180 in vaccine construct V1 showed higher fluctuations, while the side chain atoms of residues in the range 125 to 150 in vaccine construct V2 showed considerably higher fluctuations. In the case of TLR9 vaccine construct V1 and V2 complexes, the RMSF in TLR9 was slightly lower, with an average of 0.1627 nm in complex with V1, compared to the RMSF with an average of 0.2024 nm in complex with vaccine construct V2. The side chain atoms of the residues of vaccine construct V1 in complex with TLR9 showed slightly lower RMSF with an average of 0.2867 nm compared to an average of 0.3192 nm for the RMSF of side chain atoms of residues of vaccine construct V2 bound to TLR9.

#### 2.6.3. Radius of gyration evaluation

The radius of gyration (Rg) analysis for TLR3 complexes with vaccine constructs V1 and V2 showed that the Rg for TLR3 bound to vaccine construct V1 was slightly higher with an average of 3.3810 nm compared to the TLR3 bound to the vaccine construct V2 with an average of 3.2930 nm (Fig 3D). However, considerable deviations were observed in TLR3 bound to the vaccine constructs throughout the simulation period. The Rg in vaccine constructs V1 and V2 bound to TLR3 were 2.1270 and 1.9325 nm, respectively. The Rg in the TLR9 vaccine construct V1 and V2 were 3.2892 and 3.3619 nm, respectively. The Rg in TLR9 remained almost stable throughout the simulation in the case of both complexes. Meanwhile, the Rg in vaccine constructs V1 and V2 bound to TLR9 were 2.2665 and 2.1114 nm, respectively.

#### 2.6.4. Solvent accessible surface area

The buried solvent accessible surface area (B-SASA) results showed that the vaccine construct V1 had extensive interactions with the TLR9 with the resultant larger B-SASA of 21.93 nm^2^ (Fig 4A, S8 Table in S1 File). The vaccine construct V2, on the other hand, had slightly less B-SASA of 18.90 nm^2^. Both the vaccine constructs, V1 and V2, had less B-SASA in the complexes with TLR3 with B-SASA of 13.20 and 12.39 nm^2^, respectively.

**Fig 4:** The analysis of solvent accessible surface area and interaction energies. A) Total solvent aceesible surface area. Interaction energies between B) TLR3 and vaccine construct V1, C) TLR3 and vaccine construct V2, D) TLR9 and vaccine construct V1, and E) TLR9 and vaccine construct V2.

#### 2.6.5. Interaction energy analysis

The coulombic interaction energy as an electrostatic energy component, the Leenard-Jones potential energy, and the total interaction energy as a sum of coulombic and Leenard-Jones potential energy interacts were calculated between the respective vaccine constructs and TLRs. The results for the complex of TLR3 with vaccine construct V1 showed the average coulombic interaction energy of -822.76 kJ/mol with some significant deviations during the 30 to 75 ns simulation period (Fig 4B). The Leenard-Jones potential energy remained stable throughout the simulation, averaging -259.65 kJ/mol. The average total interaction energy was -1082.41 kJ/mol. Comparably, the average coulombic, Leenard-Jones, and total interaction energy was slightly higher for the TLR3 complex with vaccine construct V2 with the average of -655.58, -259.07, and -914.65 kJ/mol, respectively (Fig 4C). The coulombic interaction energy remained reasonably stable and lower throughout the simulation period for the complex of TLR9 with vaccine construct V1 with an average of -1358.94 kJ/mol (Fig 4D). The Leenard-Jones potential energy was also stable and lower, with an average of -583.30, and the total interaction energy was lowest among all the complexes under study, with an average of -1942.24 kJ/mol. Compared to the complex of TLR9 with vaccine construct V1, the complex with V2 showed slightly higher coulombic, Leenard-Jones, and total interaction energies with averages of -766.80, -493.24, -1260.04 kJ/mol, respectively (Fig 4E).

#### 2.6.6. Hydrogen bond analysis

The interchain hydrogen bonds between the TLR and vaccine constructs were analyzed. In the case of a complex of TLR3 with vaccine construct V1, an average of around 9 hydrogen bonds were formed between TLR3 residues and vaccine construct V1 residues (Fig 5, S7 Fig in S1 File). In particular, slightly more hydrogen bonds were formed during the first 50 ns simulation period, occasionally reaching a maximum of around 15 hydrogen bonds. At equilibrium, 23 hydrogen bonds were formed between the TLR3 residues and vaccine construct V1 residues. Amongst these, the hydrogen bond between TLR3 residue Asp437 and vaccine construct V1 residue Arg12 remained stable in all the studied trajectories. While, the hydrogen bonds between TLR3 residues Arg484, Glu530, Glu456, His359, Glu434, Gul456, His359, and Asn507, and vaccine construct V1 residues Cys18, Lys201, Lys120, Tyr9, Lys193, Arg197, Val13, Arg197 remained stable in multiple studied trajectories.

**Fig 5:** Hydrogen bond analysis between TLR3 and vaccine construct V1. The top panel plot the number of hydrogen bonds against simulation time. In other panels, the surface view of respective TLR (blue surface) and vaccine construct (pink surface). In the ribbon representations, the blue ribbons represent TLRs, while the orange ribbons represent vaccine constructs.

The TLR3 complex with vaccine construct V2 showed an average of around 8 hydrogen bonds during the simulation period (Fig 6, S8 Fig in S1 File). However, more hydrogen bonds were observed during the 10 to 35 ns simulation period. The trajectory of the TLR3 complex with vaccine construct V2 at equilibrium state showed 26 hydrogen bonds between TLR3 residues and vaccine construct V2 residues. Amongst these, the hydrogen bonds between TLR3 residues Lys102, Asp280, Arg222, Ser198, and vaccine construct V2 residues Glu162, Arg12, Gly110, Gly112, and Thr106 remained stable in trajectories at 25 ns, 50 ns, 75 ns, and 100 ns. Further, the trajectories at 25 ns, 50 ns, 75 ns, and 100 ns showed new and stable hydrogen bonds between TLR3 residues Tyr302, Ser198, Asn196, Glu171, Glu460, and vaccine construct V2 residues Gly16, Ser108, Gly107, and Ser22 resides.

**Fig 6:** Hydrogen bond analysis between TLR3 and vaccine construct V2. (Refer to color schemes in Fig 4).

In the TLR9 complex with vaccine construct V1, around 19 consistent hydrogen bonds were formed (Fig 7, S9 Fig in S1 File). The equilibrium trajectory showed 24 hydrogen bonds between TLR9 residues and vaccine construct V1 residues. Amongst these, the hydrogen bond between the TLR9 residues Asn263 and Glu267 and vaccine construct V1 residues Gly107, Ser181, and Ser179 remained stable in all the studied trajectories. In addition to these, the trajectories at 25 ns, 50 ns, 75 ns, and 100 ns showed a stable hydrogen bond between TLR9 residues Ala261 and Arg482 and vaccine construct V1 residues Thr106 and Ile30. While the trajectories at 25 ns, 50 ns, and 75 ns showed stable hydrogen bonds between TLR9 residues Arg426, His455, and Asp552, and vaccine construct V1 residues Glu28, Asn4, and Gly1. The hydrogen bonds between TLR9 residues Glu267, Asp259, and vaccine construct V1 residues Ser180, Ser178, and Thr106 were consistent in multiple trajectories.

**Fig 7:** Hydrogen bond analysis between TLR9 and vaccine construct V1. (Refer to color schemes in Fig 4).

In the case of the TLR9 complex with vaccine construct V2, an average of around 12 hydrogen bonds were found throughout the simulation period (Fig 8, S10 Fig in S1 File). The equilibrium state trajectory of the TLR9 complex with vaccine construct V2 showed 16 hydrogen bonds. Amongst these, the hydrogen bonds between TLR9 residues Asp453, Ser108, Gly107, and Ser22, and vaccine construct V2 residues Tyr9, Gly110, Lys8, and Cys1 remained stable in 25 ns trajectory. Further, the hydrogen bond between TLR9 residue Asp453 and vaccine construct residue Lys8 remained stable in 50 ns and 100 ns trajectories. The hydrogen bonds between TLR9 residues His531, Arg377, Arg346, Tyr321, Leu354, Thr432, Arg257, and vaccine construct V2 residues Cys1, Asp171, Gly109, Ser83, Gly111, Ser108, Glu162, Gly82, and Arg12 were observed in multiple trajectories, except the equilibrium state trajectory.

**Fig 8:** Hydrogen bond analysis between TLR9 and vaccine construct V2. (Refer to color schemes in Fig 4).

Besides the interchain hydrogen bonds, other non-bonded interactions, including salt bridges and disulfide bonds, were analyzed for each trajectory. All the trajectories of the TLR9 complex with vaccine construct V1 showed more than 200 non-bonded interactions compared to slightly fewer and more than 135 non-bonded contacts with vaccine construct V2 with TLR9. The vaccine construct V1 showed more than 60 non-bonded contacts with TLR3, while vaccine construct V2 showed more than 65 non-bonded contacts.

#### 2.6.7. Principal component analysis and Gibb’s free energy analysis

Two principal components were obtained from the covariance matrix for the backbone atoms of each complex under study. These principal components were used as reaction coordinates in analyzing Gibb’s free energy calculations. The conformations occupying positive values on PC1 and PC2 had highly correlated motions, while negative values had anti-correlating motions. The TLR3 complex with vaccine construct V1 showed two low energy basins, one between -10 to -2.5 on PC1 and -5 to 0 on PC2, and the other between 2.5 to 7.5 on PC1 and -11 to -5 on PC2 (Fig 9). On the other hand, the TLR3 complex with vaccine construct V2 showed two low energy basins, out of which one occupying the region between -12.5 to 0 on PC1 and -12.5 to 7.5 on PC2 was larger, and the one occupying the region between 16 to 21 on PC1 and -1 to 5 on PC2 was smaller. The TLR9 complex with vaccine construct V1 also showed two low energy basins, out of which the larger one occupied the region -10 to -2.5 on PC1 and -10 to 0 on PC2, and the other occupied the region 5 to 10 on PC1 and 0 to 10 on PC2. The TLR9 complex with vaccine construct V2 showed unique larger energy basins between 11 to 15 on PC1 and 0 to 5 on PC2.

**Fig 9:** Gibb’s free energy landscape. A) TLR3-vaccine construct V1 complex, B) TLR3-vaccine construct V2 complex, C) TLR9-vaccine construct V1 complex, and D) TLR9-vaccine construct V2 complex.

#### 2.6.8. Dynamic cross-correlation (DCC) analysis

The time-correlated information of inter-chain and intra-chain residue-wise contacts and motions was analyzed through DCC analysis. The vaccine construct V2 showed a stronger correlation between the first 25 residues of V2 and around the first 450 residues of TLR3 (Fig 10). Meanwhile, the vaccine construct V1 showed a slightly weaker correlation between the first 25 residues of V1 and TLR3 residues in the range of 200–650. The first 25 residues of vaccine construct V2 in the TLR9 complex also showed a strong correlation with the residues of TLR9 in the range 200–400. The vaccine construct V1 showed a slightly weaker correlation with TLR9 residues in the range of 50–400.

**Fig 10:** DCC analysis for A) TLR3-vaccine construct V1 complex, B) TLR3-vaccine construct V2 complex, C) TLR9-vaccine construct V1 complex, and D) TLR9-vaccine construct V2 complex.

#### 2.6.9. MM-GBSA calculation

The MM-GBSA calculations were performed on 500 trajectories with the lowest energy conformations sampled from the larger energy basins of each TLR vaccine construct complex. The MM-GBSA calculations were carried out, taking into account the entropic energies. The results of MM-GBSA calculations are shown in Table 5. The respective vaccine construct’s binding affinity (ΔGbinding) was calculated from the entropic energy and electrostatic, polar and nonpolar solvation energies from the van der Waals. The vaccine construct V2 showed the lowest and most favorable ΔG_binding_ of -159.60 kcal/mol in complex with TLR3.

**Table 5:** MM-GBSA calculations for TLR and vaccine constructs.

Energy component (kcal/mol)	Vaccine construct V1		Vaccine construct V2	
	TLR3	TLR9	TLR3	TLR9
Entropy (-TΔS)	21.42 (2.79)	21.50 (0.05)	15.78 (0.05)	27.26 (0.35)
ΔVDWAALS	-78.04 (7.65)	-80.88 (16.11)	-177.45 (12.92)	-153.69 (13.06)
ΔEEL	-692.27 (19.61)	-523.47 (23.76)	52.08 (13.29)	24.78 (18.04)
ΔEGB	697.59 (20.18)	539.74 (17.27)	-36.86 (17.63)	-6.64 (11.44)
ΔESURF	-12.76 (0.72)	-10.69 (0.87)	-23.24 (0.57)	-22.47 (1.26)
ΔGGAS	-770.31 (23.64)	-604.35 (30.19)	-125.37 (21.89)	-128.91 (25.89)
ΔGSOLV	684.83 (20.19)	529.04 (17.30)	-60.11 (17.64)	-29.11 (11.51)
ΔTOTAL	-85.48 (31.09)	-75.30 (34.79)	-185.48 (28.12)	-158.02 (28.33)
ΔG_binding_	-56.00 (9.31)	-45.28 (8.62)	-159.60 (9.56)	-111.59 (12.44)

ΔVDWAALS: van der Waals energy; ΔEEL: Electrostatic energies; ΔEGB: Polar solvation energy; ΔESURF: Nonpolar solvation energy; ΔGGAS = ΔVDWAALS+ΔEEL; ΔGSOLV = ΔEGB+ ΔESURF; ΔTOTAL = ΔGSOLV +ΔGGAS; ΔG_binding_ = ΔTOTAL−TΔS. (Standard deviations are given in parentheses)

In contrast, the vaccine construct V1 showed significantly higher and comparably less favorable ΔG_binding_ of -56.00 kcal/mol in complex with TLR3. In the case of TLR9 complexes, the vaccine construct V2 showed lower and favorable ΔG_binding_ of -111.59 kcal/mol, compared to the ΔG_binding_ of -45.28 kcal/mol for the vaccine construct V1. The vaccine construct V2 showed the lowest van der Waal’s energies (ΔVDWAALS) of -177.45 and -153.69 kcal/mol for TLR3 and TLR9, respectively. Meanwhile, van der Waal’s energies were significantly higher in the case of vaccine construct V1 in complex with TLR3 with energies of -78.04 and -80.88 kcal/mol, respectively. The electrostatic energies (ΔEEL) were positive and significantly higher for the vaccine construct V2 than the vaccine construct V1 in complex with TLRs. While the polar solvation energies (ΔEGB) were significantly lower for the complexes with vaccine construct V2 than the vaccine construct V1.

### 2.7. Immune simulation studies

According to the results of the immuno simulation study, the vaccination may generate a general immune response that is in line with the body’s natural defences. Moreover, an increases in the host’s concentrations of helper T cells, cytotoxic T cells, plasma B cells, and active B cells were found, suggesting the development of an incredibly strong immune response and memory of immunisation in addition to increased antigen clearance. The vaccination can produce an amazing variety of different types of cytokines, including interleukin-23, interferon-γ, IL-10, and IFN-β, which are essential for eliciting an immune response and protecting the body against viruses. All in all, the immune simulation study revealed that the vaccine has a number of intriguing properties that could lead to strong immune responses in the host once it is administered. The figure is presented in S11 Fig in S1 File.

## 3. Discussion

Cryptococcosis, a lethal mycosis, is instigated by the pathogenic species *C*. *neoformans* and *C*. *gattii*, primarily affects the lungs, manifesting as pneumonia, and the brain, where it presents as meningitis. It poses a grave threat, especially to immunocompromised individuals like HIV patients, leading to severe neurological complications. Mortality rates can reach 100% if untreated, emphasizing the urgent need for effective management strategies and awareness [1, 13]. As opposed to conventional immunization techniques, epitope-based vaccines have a number of benefits, including high specificity, extended efficiency, improved safety, simplicity in manufacturing and storage, and the capacity to target epitopes that can concurrently protect against *C*. *neoformans* and *C*. *gattii* [24, 25]. Consequently, this work used immunoinformatics and extended dynamics simulations to create and validate two multiepitope polyvalent vaccines that target the pathogenic proteins of *C*. *neoformans* and *C*. *gattii*. Two proteins, Chaperone DnaK and Heat shock transcription factor, were selected from both *C*. *neoformans* and *C*. *gattii* for their fundamental roles in gene expression regulation, protein stability maintenance, and cellular integrity, especially under stress conditions [5, 22]. Obtained from UniProt, their sequences were selected for vaccine development due to their anticipated antigenicity and favorable physicochemical characteristics.

Utilizing these proteins, epitope mapping was able to detect CTL, HTL, and LBL epitopes all crucial for enhancing the host’s defenses against viral infection. The vaccine formulation was chosen based on highly antigenic, non-allergenic, and non-toxic epitopes, demonstrating their ability to trigger a healthy immune response against viral infection, using IEDB algorithms. High standards for antigenicity, non-allergenicity, non-toxicity, and, in the case of HTL epitopes, the capacity to elicit at least one cytokine response were used to select 8 CTL, 8 HTL, and 8 LBL epitopes. Finally, utilizing EAAAK, AAY, GPGPG, and KK linkers at the proper locations, the best chosen epitopes were linked to develop two vaccine constructions, V1 and V2. To boost their immunogenicity in the human body, the PADRE sequence and hBD adjuvants were also linked. While the PADRE sequence was used as an immunostimulant to boost vaccination efficiency, the hBD adjuvant strengthened host defense by drawing immature dendritic cells, naïve memory T cells, and monocytes toward the infection site. Linkers were included to stabilize the vaccine design and increase antigenicity, and EAAAK inhibits vaccine degradation [26–30].

Both vaccine constructs showed high antigenic scores, with V1 at 2.0334 and V2 at 1.8471, much higher than the 0.6182 score reported in a similar vaccine study targeting a different fungal pathogen. These higher scores suggest a greater ability to elicit a robust immunological response, confirming the enhanced efficacy. These superior scores suggest an enhanced potential to induce a robust immune response, confirming the efficacy of our constructs. Additionally, both vaccine designs displayed non-allergenicity and non-toxicity, indicating their safety profile and reinforcing their suitability for further development. Furthermore, it was shown that both constructs were soluble, scoring 0.820 for V1 and 0.809 for V2 in the vaccine solubility index. These values are nearly on par with the 0.829 score of the comparable vaccine, highlighting that our constructs exhibit a similar and effective level of solubility [31–33]. An insoluble vaccine entails the risk of both inefficiency and tangled peptide aggregates accumulation in the body. As solubility is an important aspect of these two vaccine constructions, any solubility index above 0.45 indicates a higher level of solubility [34, 35]. The physicochemical property study demonstrated the competency of the vaccination constructs. A vaccination is said to be stable if its instability index is less than 40, and unstable if it is greater than 40 [36]. Both vaccination constructs were stable, with instability indexes of 27.67 and 30.82 for vaccine constructions V1 and V2, respectively. The vaccines indicated to be stable at normal human body temperature based on the aliphatic index values of 56.26 and 64.09 for vaccine constructs 1 and 2, respectively, which measures thermostability [37]. Both vaccines exhibit a negative GRAVY value, with values of -0.419 and -0.376 respectively. This negative value indicates their hydrophilicity, suggesting their enhanced solubility in water [38]. Furthermore, the vaccine contains numerous pairs of amino acids that may be mutated into cysteine residues, increasing the vaccine’s durability and effectiveness, according to disulfide engineering of the vaccine designs.

Secondary structure analysis revealed that a random coil was the most prevalent structure in the vaccination prototypes. In order to confirm the validity of the vaccination models after the tertiary structure prediction, the ERRAT and Ramachandran plots were assessed. A model exhibiting a score of greater than 50 on the ERRAT, which stands for overall quality factor, is considered to be of high quality [39]. The models of the vaccine constructions demonstrated notable ERRAT scores of 96.744 and 96.190, indicating excellent quality. The Ramachandran plot, where the majority of residues should ideally lie within the favored region, is a method for assessing the accuracy of predicted protein structures [40]. A significant fraction of residues for both vaccine designs (92.0% for vaccine construct-1 and 93.1% for vaccine construct-2) were found to dwell inside this favored region, according to analysis of the Ramachandran plot. Both vaccine designs have desirable characteristics and structures, and they should be stable enough, according to the results of the overall biophysical and structural prediction study.

Through molecular docking study with the ClusPro 2.0 and HDOCK Server, the interaction between the two vaccine constructs and TLR2 (PDB ID: 2z80), TLR3 (PDB ID: 2a0z), and TLR9 (PDB ID: 3wpf) was evaluated. An important determinant of effective infection control is the relationship between vaccines and TLRs. TLRs serve an important role in triggering an adequate immune response. TLR2, TLR3, and TLR9 have been recognised as possible targets for the Cryptococcus vaccine. TLR2 and TLR3 has the capability to identify multiple ligand and both are involved in infection and recognition of Cryptococcal infection via increasing pro-inflammatory cytokines. TLR9 has the ability to detect fungal genomic DNA and recognise the unmethylated CpG motifs of C. neoformans, which results in the recruitment of phagosomes and the removal of the fungal pathogen [41, 42].

By targeting these TLRs, Cryptococcus vaccines can stimulate both innate and adaptive immune responses, leading to improved protection against both *C*. *neoformans* and *C*. *gattii* infection. Both vaccine constructs exhibited strong affinity with all three TLRs studied. During the docking analyses conducted with ClusPro and HDock server, a markedly negative score indicates robust binding affinity [43]. Vaccine construct-V1 demonstrated the strongest binding affinity with TLR9 (-1245.5) in the ClusPro analysis and with TLR3 (-306.03) in HDock. Conversely, vaccine construct-V2 exhibited significant binding with TLR3 (-1040.1) in the ClusPro analysis and the highest affinity with TLR9 (-297.61) in HDock server. A previous study having the similar TLRs showed relevant outcomes, where vaccine construct 1 showed the highest binding score with TLR9 (-1337.7 Kcal/mol) and vaccine construct 2 exhibited strongest affinity against TLR3 (-1290.8 kcal/mol) [21].

The docked complexes of TLR3 with vaccine constructs V1 and V2 and TLR9 with vaccine constructs V1 and V2 were subjected to 125 ns MD simulations to delve deeper into the stability of respective complexes and gauge the binding affinity of respective vaccine constructs. The analysis of RMSD provides valuable insights into the overall stability of the systems under a biologically relevant environment [44], where the structural deviations in backbone atoms from the starting equilibrated structure are measured. The RMSF analysis provides valuable insights into the flexibility of side chain atoms of residues [45, 46], which might result in secondary structural changes and adaptation to stable and rigid conformations. While the Rg analysis provides insights into the overall compactness of the structure [47], where higher Rg indicates the unfolding event in the protein structure. The TLR structures are unique because they contain structural motifs known as leucine-rich repeat (LRR) of around 22–29 residues containing beta-strands and alpha-helices [48]. TLR3 and TLR9 are transmembrane proteins and contain 670 and 781 residues, respectively. Both TLRs possess a unique horseshoe-shaped structure conferring rigidity and stability and a unique structure where a structural motif of vaccine or pathogen-associated molecular patterns can bind [49].

The RMSD in TLR9 compared to TLR3 indicated better stability with subtle deviations, whereas TLR3 has a higher magnitude of deviations throughout the simulation period. Both the vaccine constructs almost equally augmented the stability of TLR9 in terms of RMSD, whereas vaccine construct V1 seems to stabilize the TLR3 better compared to vaccine construct V2.

The fluctuations in side chain atoms of TLR9 bound to vaccine construct V1 or V2 further confirm the stability where most of the residues had lower than 0.3 nm RMSF, while the residues in the range 425 to 500 from the central loop region show reasonable and obvious flexibility. While around 100 residues in each terminal end and central loop-rich region of TLR3 are quite flexible and have considerable fluctuation in terms of higher RMSF. The RMSF in vaccine construct V2 is relatively stable compared to vaccine construct V1. Both the vaccine constructs are 247 residues long but differ in the structured regions where vaccine construct V2 assumes more α-helices and β-sheets and fewer loop regions, which shows higher RMSF in loop residues in the range of 125–150. The vaccine construct V1 has fewer structured regions and more loops, which might have resulted in considerable fluctuations in the side chain atoms of loop residues in the ranges 60–80, 120–140, and 160–170. However, the RMSF in both vaccine constructs remained lower in the complex with TLR9, indicating that the complexes with TLR9 are more stable than TLR3.

The Rg analysis further confirms the stability of TLR9 structures in complex with both vaccine constructs. However, vaccine construct V2 restricts the rotation of TLR9 around its axis and confers better stability than vaccine construct V1. In the case of TLR3, Rg suggests a slightly less stable structure, possibly due to the extended loop region located centrally in TLR3. In TLR3, the vaccine construct V2 stabilizes the structure of TLR3 better than vaccine construct V1. The Rg in vaccine construct V2 bound to TLR3 and TLR9 is more stable than vaccine construct V1.

The buried solvent-accessible surface area (B-SASA) is the portion of SASA that becomes inaccessible when the vaccine construct binds to the TLR to form the complex of TLR with the vaccine construct. The higher the B-SASA, the more the surface area of the vaccine construct is in contact with the TLR. Consequently, it can make better interactions, resulting in better binding affinity. Vaccine construct V1 has almost twofold B-SASA in the complex with TLR9 compared to TLR3. Meanwhile, the vaccine construct V2 has slightly lower B-SASA in both complexes. The vaccine construct V1 indicates strong binding affinity due to more exposed surface area and, consequently, more interactions.

The interaction energy analysis revealed that the vaccine construct V1 has a significantly stable and favorable coulombic interaction energy and relatively stable Leenard-Jones potential energy. The total interaction energy result is significantly lower and favorable for vaccine construct V1 in the complex with TLR9 among all the complexes. The vaccine construct V2 having better and favorable interaction energies for the TLR9 further suggests that both the vaccine constructs have better binding affinities against the TLR9.

The interchain hydrogen bonds are important in the stability of the protein-protein complex [50], and the more interchain hydrogen bonds, the better the resulting protein-protein complex [51]. A comparably higher number of interchain hydrogen bonds in TLR9 with vaccine construct V1 indicates stronger stability than its complex with TLR3. The vaccine construct V2 also had a reasonably good number of interchain hydrogen bonds with TLR9 compared to TLR3. TLR9 complexes with vaccine construct V1 and V2 further suggest few consistent hydrogen bonds throughout the simulation period. Apart from the hydrogen bonds other non-bonded interactions key clearly indicates that the vaccine construct V1 has more number of non-bonded interactions with TLR9 compared to vaccine construct V2. However, slightly less number of non-bonded interactions between vaccine constructs V1 and V2 with TLR3 suggests lower stabilizing propensity of these vaccine constructs against TLR3.

The PCA analysis and Gibb’s free energy estimates indicate that the TLR3 complex with vaccine construct V2 has many lower energy metastable conformations than the TLR3 complex with vaccine construct V1. While the TLR9 complex with the vaccine construct V1 has more low energy conformations than the TLR9 complex with vaccine construct V2. The DCC analysis further confirms more positively correlated residue-residue contacts between TLR9 and vaccine construct V1 and V2 compared to TLR3 complexes. In the case of TLR3 complexes, through strong positively correlated residue-residue contacts, there are evident that there are more negatively correlated residue-residue contacts, which might be responsible for slightly lower stability of corresponding complexes compared to TLR9 complexes.

The MM-GBSA calculations, considering the entropic energies and other energies such as van der Waals, electrostatic, polar solvation, and solvent-accessible surface area energy, give valuable insights into the binding affinities [52]. The sampling of trajectories can have a significant effect on the ΔG_binding_ calculation. Hence, the lowest energy conformations sampled from Gibb’s free energy landscape are biologically more relevant and can give a more accurate measure of ΔG_binding_. The vaccine construct V2 exhibited a stronger binding affinity for the TLR3 than TLR9 and an almost twofold better affinity than the vaccine construct V1 against TLR3 and TLR9. The results also support the interaction energy analysis where the vaccine construct V2 has the lowest coulombic and Leenard-Jones interaction energies.

This computational approach concluded a vaccine candidate with high potential to target both Cryptococcus neoformans and Cryptococcus gattii. While these in silico results are very encouraging, we recognize that the ultimate validation of any vaccine candidate is experimental confirmation, which is required to prove efficacy and safety thoroughly. However, due to present limitations in access to sophisticated laboratory equipment and a lack of appropriate animal models, we could not conduct wet lab studies or in vivo trials as part of this investigation. These limits, while unfortunate, highlight the significance of future experimental efforts to validate and expand on our computational findings. We recommend synthesizing the identified epitopes and conducting in vivo studies to validate the vaccine’s efficacy, in order to progress beyond computational predictions. These steps are crucial for transitioning the computational predictions into a validated and effective vaccine candidate, which could be more efficient than traditional vaccines.

## 4. Methods

The stepwise methodology of the entire study is depicted in S12 Fig in S1 File as a flowchart.

### 4.1. Selection of proteins and physicochemical property analyses

Virulent proteins for *C*. *neoformans* and *C*. *gattii* named Chaperone DnaK and Heat shock transcription factor were selected for the study. The target protein sequences were then retrieved in FASTA format from the UniProt database (https://www.uniprot.org). In order to evaluate the antigenic property, the selected protein was analyzed in the online antigenicity tool VaxiJen v2.0 (http://vaxijen/VaxiJen/VaxiJen.html). Based on auto cross covariance (ACC) translation of protein sequences into uniform vectors of principal amino acid characteristics, vaxijen offers an alignment-free method for antigen prediction. Transmembrane topology was analysed employing the TMHMM-2.0 server (https://services.healthtech.dtu.dk/service.php?TMHMM-2.0).). TMHMM is a hidden Markov model-based approach for predicting membrane protein topology, identifying transmembrane helices, and discriminating between soluble and membrane proteins. By utilizing the ExPASy ProtParam server (https://web.expasy.org/protparam//), We investigated many physicochemical properties of the proteins.

### 4.2. Epitope mapping and construction of vaccine

The online epitope prediction server Immune Epitope Database (IEDB; https://www.iedb.org/), was used to determine the T-cell and B-cell epitopes of the chosen protein sequences. all the parameters kept at default setting during prediction. The MHC class I-restricted CD8+ cytotoxic T-lymphocyte (CTL) epitopes of the chosen sequences for a few prevalent human leukocyte antigen (HLA) alleles (i.e., HLA A_01:01, HLA A_02:01, HLA A_02:06, HLA A_03:01, HLA A_11–01, and HLA A_29:02) were predicted using the suggested NetMHCpan EL 4.0 prediction method (http://tools.iedb.org/mhci/), maintaining the length of the epitopes at 9 (9-mer epitopes). Likewise, we identified the MHC class II-restricted CD4+ helper T-lymphocyte (HTL) epitopes for a few common HLA alleles (DRB1_03:01, DRB1_04:01, DRB1_15:01, DRB5_01:01, DRB4_01:01, and DRB3_01:01) by employing the 2.22 prediction method, under the IEDB (http://tools.iedb.org/mhcii/), while maintaining a 15-mer epitope length. The BepiPred linear epitope prediction technique 2.0 was used to predict the Linear B Lymphocytes (LBL) of the specified proteins while keeping all of the default values. The top-scored LBL epitopes with more than ten amino acids were determined to be viable candidates for additional investigation based on this study [21, 53].

We used the VaxiJen v2.0 server to identify epitope antigenicity, the TMHMM 2.0 server to predict transmembrane topology, and to evaluate allergenicity we used the AllergenFP (https://ddg-pharmfac.net/AllergenFP/) and AllerTOP (https://www.ddg-pharmfac.net/AllerTOP/) and AlgPred2.0 (https://webs.iiitd.edu.in/raghava/algpred2/ige.html) server. Additionally, we used the ToxinPred server (http://crdd.osdd.net/raghava/toxinpred/) to assess toxicity. ToxinPred employs a Basic Local Alignment Search Tool-based approach, as well as similarity and motif-based techniques, to obtain a significant probability of successful prediction despite low sensitivity. The potential of the HTL epitopes to elicit IFN-g, IL-4, and IL-10 was anticipated employing the IFNepitope (http://crdd.osdd.net/raghava/ifnepitope/), IL4pred (http://crdd.osdd.net/raghava/il4pred/), and IL10pred (http://crdd.osdd.net/raghava/IL-10pred/) servers, accordingly [54–56]. Furthermore, the conservation of the epitopes was assessed using the IEDB epitope conservancy tool (http://tools.iedb.org/conservancy/). Epitopes having the greatest potential for vaccine development were selected according to their exceptional antigenicity, non-toxicity, non-allergenicity, and conservancy. The adjuvants PADRE and human beta-defensin (hBds), as well as the selective linkers EAAAK, AAY, GPGPG, and KK, have been incorporated with these epitopes to generate the vaccine [30, 57, 58].

### 4.3. Analyses of the biophysical and structural properties of the vaccine

Antigenicity and allergenicity investigations were performed to guarantee that the vaccine was safe and effective. The Protein-Sol server (https://protein-sol.manchester.ac.uk/) was used to determine the solubility of the vaccine design when expressed in Escherichia coli. Protein-Sol predicts protein solubility from Escherichia coli cell-free expression data by computing 35 sequence-based features and assigning feature weights to low and high solubility subgroups. The ProtParam tool of the ExPASy server was used to examine the biophysical properties of the vaccine constructs, such as isoelectric pH, aliphatic and instability index, GRAVY values, hydropathicity, expected half-life, and other features. Two servers, SOPMA (https://npsa-prabi.ibcp.fr/cgi-bin/npsa_automat.pl?page=/NPSA/npsa_sopma.html) and PSIPRED (http://bioinf.cs.ucl.ac.uk/psipred/), were used to predict the secondary structure of the final vaccine [59, 60]. The tertiary structure of the vaccine constructs was modulated using the trRosetta server (https://yanglab.nankai.edu.cn/trRosetta/), and subsequently refined using the GalaxyRefine module of the GalaxyWEB server (http://galaxy.seoklab.org/). The trRosetta server is a web-based tool for protein structure prediction that uses deep learning and Rosetta to predict inter-residue geometries and translate them into constraints, guiding structure prediction via direct energy minimisation. The enhanced models were verified using the ProSA-web server (https://prosa.services.came.sbg.ac.at/prosa.php) for Z score plots and the PROCHECK server (https://saves.mbi.ucla.edu/) for Ramachandran and ERRAT score plots [61–64].

### 4.4. Disulfide engineering of the vaccine construct

To study the structural stability of folded proteins, vaccine protein disulfide engineering was carried out utilising the Disulfide by Design 2 server (http://cptweb.cpt.wayne.edu/DbD2/). During the examination, the Cα-Cβ-Sγ angle maintained at 114.6° ± 10, whereas the χ3 angle was adjusted at -87° or +97. The process of creating disulfide bridges involved selecting pairings of residues with energy less than 2.5 Kcal/mol and converting them to cysteine residues [65].

### 4.5. Molecular docking

To anticipate the binding intensities and interaction patterns of the vaccine constructs with the TLR2 (PDB ID: 2z80), TLR3 (PDB ID: 2a0z), and TLR9 (PDB ID: 3wpf) receptors, molecular docking study was performed. The mutant 3D structure of the multi-epitope construct functioned as the ligand, whereas the RCSB PDB database provided the TLR2, TLR3, and TLR9 receptor structures, which were prepared by BIOVIA Discovery studio. HDOCK Server (http://hdock.phys.hust.edu.cn) and ClusPro 2.0 were used to calculate the binding affinity between the vaccine construct and TLRs [43, 66]. ClusPro server characterizes docked models by the centers of densely packed clusters of low-energy structures and hdock server efficiently anticipates their interaction using a hybrid approach of template-based and template-free docking. ClusPro and HDOCK were chosen for our docking study because of their demonstrated reliability and broad use in related studies. Several investigations show that both servers frequently generate reliable results in protein-protein and protein-ligand docking. Additionally, we compared the docking results of our complexes with TLR complexes that were previously characterized in order to further validate the docking approach [21, 43]. Pymol software was utilized to visualize the interactive residue between vaccine and TLR complex. The least energy-weighted score and docking efficiency were used to determine the best-docked complex.

### 4.6. Molecular dynamics simulation

The docked complexes of TLR3 and TLR9 with respective vaccine constructs V1 and V2 were selected for the MD simulations. The MD simulations extending up to 125 ns were performed using the Gromacs 2020.4 [67] program on the HPC cluster at Bioinformatics Resources and Applications Facility (BRAF), C-DAC, Pune. Initially, the topologies of respective proteins from the four complexes *viz*. TLR3-vaccine construct V1 (TLR3-V1), TLR3-V2, TLR9-V1, and TLR9-V2 were built with CHARMM-36 force field parameters [68, 69]. Each complex was solvated with TIP3P water model [70] in a box of dodecahedron unit cells, which were placed, keeping the system’s boundary 1 nm away from its edges. The resulting systems were neutralized with 0.15 molar concentration of NaCl. The neutralized systems were further energy minimized by employing the steepest descent algorithm where the force constant threshold was set to 100 kJ mol^-1^ nm^-1^. The equilibration was performed in two stages. The first equilibration was performed at constant volume and constant temperature (NVT) conditions for 1 ns, where the temperature of 300 K was achieved with modified Berendsen thermostat [71]. The second equilibration was performed at constant volume and constant pressure (NPT) conditions for 1 ns, where 1 atm pressure was achieved with Berendsen barostat [72]. The unrestrained production phase MD simulations of 100 ns were performed on each equilibrated system where the temperature was held constant with a modified Berendensen thermostat and pressure was held constant with the Parrinello-Rahman barostat [73]. However, the covalent bonds were restrained with the LINCS algorithm [74]. The long-range electrostatic energies at 1.2 nm cutoff distance were computed with the Particle Mesh Ewald (PME) method [75]. The stability of each system was analyzed in terms of the root mean square deviations (RMSD) from the initial equilibrated positions of backbone atoms of TLR chains as well as the respective vaccine chains.

Similarly, the fluctuations in the side chain atoms of TLR and vaccine chains were analyzed as root mean square fluctuation (RMSF). The compactness of the system during MD simulation was analyzed in terms of radius of gyration (Rg). The affinity of respective vaccine constructs against TLR3 or TLR9 was analyzed in terms of the number of hydrogen bonds formed. The residues involved in hydrogen bond formation as well as other non-bonded interactions were interpreted at different time intervals of MD simulation.

Further, the buried solvent-accessible surface area (B-SASA) was calculated to get insights into the shared SASA by the respective TLRs and the vaccine components [76, 77]. In the SASA analysis, the SASA was calculated separately for the TLRs, vaccine components, and the TLR vaccine complexes. The buried solvent accessible surface area was calculated through Eq (1).

$$B-SASA\;\left({nm}^{2}\right)=0.5\left({SASA}_{TLR}+\;{SASA}_{vaccine\;component}-{SASA}_{TLR-Vaccine\;complex}\right).$$ (1)

Where B-SASA is buried solvent accessible surface area shared between TLR and vaccine component, SASA_TLR_, SASA_vaccine component_, and SASA_TLR-vaccine complex_ are the total solvent accessible surface areas of TLR, vaccine component, and TLR vaccine complex, respectively.

The total interaction energies between TLRs and respective vaccine components were calculated from the Coulombic interaction energy and Leenard-Jones potential energy between the TLR and vaccine components.

The dominant path of motions in corresponding TLR vaccine complexes were analyzed from principal component analysis (PCA) [78], where the covariance matrix for the backbone atom of each complex was obtained from the gmx covar program. After diazonalizing this covariance matrix, the eigenvectors and eigenvalues were obtained. Eigenvectors or principal components showed the path of motion, while the eigenvalues showed the mean square fluctuation. The first two principal components (PC1 and PC2) were used as a reaction coordinates in analyzing the Gibb’s free energy surfaces [79] with gmx sham program. Dynamical cross-correlation matrix (DCCM) [80] analysis was performed to analyze the extent to which the fluctuations and displacements of side chains of each TLR chain and vaccine chain are correlated with one another. In the DCC plots, the color gradient ranges from blue (negative correlation, less likely) to red (positive correlation, more evident), corresponding to the correlation coefficients -1 and +1, respectively, and the lighter shades indicate weaker correlations where the white color indicates no correlation.

The end state free energy calculations employing the Molecular mechanics with generalised Born and surface area solvation (MM-GBSA) method [81] were performed. The sampling of trajectories used in MM-GBSA calculations significantly influences the binding affinities. The MM-GBSA calculations were performed on 500 trajectories extracted from the lowest energy basins identified from Gibb’s free energy landscape analysis. The binding affinities in terms of ΔG_binding_ in kcal/mol were calculated considering the entropic contributions.

The protein structures were rendered in ChimeraX [82], PyMOL [83], and VMD [84], and graphs were plotted in the XMGRACE [85] interface. The hydrogen bond interaction network diagrams between TLR and vaccine constructs were generated using a standalone PDBSUM program [86]. Gibb’s FEL plots were generated using the Python-based Matplotlib package [87], while the DCCM analysis was performed in the R statistical program [88] using the Bio3D package [89].

### 4.7. Immune simulation studies

The C-ImmSim internet server (http://150.146.2.1/C-IMMSIM/index.php), which offers real-time immune interaction prediction, was used to carry out the immunological simulation of the vaccine. All parameters were kept at default, except for the time steps, which were set at 1, 84, and 170, and the number of simulated steps, which was set at 1,050. The suggested dosage for the vaccination is three injections every four weeks, which corresponds with the intervals between doses that should be followed for all commercial vaccines [90, 91].

## 5. Conclusion

In this study, we utilized an integrated bioinformatics approach to design a polyvalent multiepitope subunit vaccine targeting the virulent proteins Heat Shock Transcription Factor and Chaperone DnaK of *C*. *neoformans* and *C*. *gattii*. The vaccine constructs developed through epitope prediction, molecular docking, and molecular dynamics simulations exhibited strong antigenicity, stability, non-toxicity, and favorable interactions with TLRs, particularly TLR9. The molecular dynamics simulations and MM-PBSA binding free energy calculations further confirmed the stability and binding affinity of Vaccine Construct V1. These findings offer a promising foundation for the development of an effective cryptococcal vaccine. Given the urgent need for novel therapeutic options for cryptococcosis, this study represents a significant step towards a potential preventive measure against this life-threatening fungal infection. Future in vivo studies are essential to validate the immunogenicity and protective efficacy of these vaccine constructs, thereby advancing the prospects of their clinical application.

## Supporting information

S1 File Tables & figures. (DOCX)
